# A Systematic Review on Selected Complications of Open-Wedge High Tibial Osteotomy from Clinical and Biomechanical Perspectives

**DOI:** 10.1155/2021/9974666

**Published:** 2021-10-31

**Authors:** Elaheh Elyasi, Guillaume Cavalié, Antoine Perrier, Wilfrid Graff, Yohan Payan

**Affiliations:** ^1^Univ. Grenoble Alpes, CNRS, TIMC-IMAG, 38000 Grenoble, France; ^2^Service de Chirurgie Orthopédique et Traumatologie, Site Nord., CHU Grenoble-Alpes, La Tronche, France; ^3^Univ. Grenoble Alpes, Laboratoire d'Anatomie des Alpes Françaises, Domaine de la Merci, 38700 La Tronche, France; ^4^Service de Chirurgie Osseuse et Traumatologique, Centre de Référence Des Infections Ostéo-Articulaires Complexes, Groupe Hospitalier Diaconesses–Croix Saint-Simon, 125, Rue d'Avron, 75020 Paris, France

## Abstract

**Background:**

The wedge opened during high tibial osteotomy defines the alignment correction in different body planes and alters soft tissue insertions. Although multiple complications of the surgery can be correlated to this, there is still a lack of consensus on the occurrence of those complications and their cause. The current study is aimed at clarifying this problem using a combined medical and biomechanical perspective.

**Methods:**

We conducted a systematic review of the literature on selective complications of the surgery correlated with the angles of the opened wedge. Search topics covered tibial slope alteration, patellar height alteration, medial collateral ligament release, and model-based biomechanical simulations related to surgical planning or complications. *Findings*. The selection process with the defined inclusion/exclusion criteria led to the collection of qualitative and quantitative data from 38 articles. Medial collateral ligament tightness can be a valid complication of this surgery; however, further information about its preoperative condition seems required for better interpreting the results. The posterior tibial slope significantly increases, and the patellar height (using the Blackburne-Peel ratio) significantly decreases in the majority of the selected studies. Model-based biomechanical studies targeting surgical planning are mostly focused on the lower-limb alignment principles and tibiofemoral contact balancing rather than surgical complications. *Interpretation*. Increased posterior tibial slope, patellar height decrease, and medial collateral ligament tightness can occur due to alterations in different body planes and in soft tissue insertions after wedge opening. This study clarified that information about preoperative alignment in all body planes and soft-tissue conditions should be considered in order to avoid and anticipate these complications and to improve per surgery wedge adaptation. The findings and perspective of this review can contribute to improving the design of future clinical and biomechanical studies.

## 1. Introduction

Open-wedge high tibial osteotomy (OWHTO) is a joint preserving treatment for medial knee osteoarthritis used especially for young and active patients with a varus deformity [1–3]. The purpose of this surgery is to transfer the excessive axial loads applied on the medial compartment of the knee to the lateral compartment. This can be achieved by performing a wedge osteotomy on the medial side of the proximal tibia that results in moving the mechanical axis of the lower limb to pass through the lateral tibiofemoral compartment rather than the medial compartment [4, 5].

The main difficulty of this surgery is to find the correct modification of limb alignment that significantly reduces the pressure and contact area of the medial compartment without increasing these values in the lateral compartment or creating laxity in valgus. The amount of the required correction is traditionally defined based on the frontal projected X-ray. In these cases, the patient's X-ray is used to define the weight-bearing axis (WBA) or the standing hip–knee–ankle (HKA) angle, and the surgeon decides on the correction amount based on a recommended zone that has been suggested by the literature for either of these parameters [6–8]. However, these protocols do not seem to be the optimum solution for all the patients because the follow-up studies show a high rate of under or overcorrected cases [5] with deterioration of the outcomes in longer follow-ups [9, 10]. The unsolved question of realignment has resulted in multiple studies taking various approaches including clinical studies [11, 12] and in vivo or cadaveric biomechanical studies [13, 14]. However, there is still a high lack of consensus on the ideal alignment after HTO, and some study results even seem to be contradictory.

From a biomechanical perspective, the exact size and shape of the wedge opened on the tibia during the osteotomy process define the amount of alteration made on the lower limb alignment not only in the frontal plane but also in the sagittal plane. In addition to that, the angles of the opened wedge can be directly related to the change of tension inside the soft tissues whose insertion site has been altered during HTO. D'Entremont et al. performed a study using a magnetic resonance imaging (MRI) based method on OWHTO and found that this surgery changes both tibiofemoral and patellofemoral kinematics in a manner that cannot be assessed using conventional radiology [15]. As a result, it seems necessary to take a different perspective while analyzing the complications of OWHTO and trace the complications that could have been caused by having a simplistic view of wedge opening during the planning step.

Nonconsideration of changes in the sagittal plane during the planning step can lead to alteration of the tibial slope [16]. Some observations show that increased posterior tibial slope can induce an anterior translation of the tibia with respect to the femur which opens a concern about whether it can increase the strain of the anterior cruciate ligament (ACL) and result in a higher risk of ACL rupture [17]. On the other hand, change of tension inside the soft tissues whose insertion site has been altered during OWHTO can be traced to complications such as increased pressure in the medial tibiofemoral compartment due to medial collateral ligament (MCL) tightness [18]. This effect of alteration in a soft tissue insertion can also be correlated to the alteration in the position of the patella as it is attached to the patellar tendon. The exact clinical effect of alteration in patellar position is still unclear on patellofemoral pain, but symptoms of association with patellofemoral pain have been observed with patellar lateral shift [19] and also observation of patellofemoral arthritis in second-look arthroscopy [20]. While the aforementioned complications can be foreseen from a biomechanical point of view, their occurrence may be still a place of debate among different clinical and cadaveric studies with contradictory results.

As a result, the objective of this systematic literature review is to investigate the occurrence of tibial slope alteration, patellar position modification, and excessive pressure due to MCL tightness after OWHTO and to discuss their sources and correlation with the opened wedge angles. In this context, the medical literature is considered as a starting point while at the discussion level, a biomechanical perspective is also added to assist the interpretation of the results. Finally, model-based biomechanical studies targeting the planning of HTO are also addressed to find out their role in better distinguishing the parameters involved in the surgery.

## 2. Methods

### 2.1. Search Strategy

We performed a systematic literature review through PubMed, Science Direct, and Cochrane in accordance with the PRISMA protocol. The last bibliographic search was done on November 20, 2019. The electronic search strategy developed by the authors was critically reviewed by a health science librarian, using the guideline statement of Peer Review of Electronic Search Strategies (PRESS) 2015 [21]. The search concepts included (1) studies addressing suboptimal outcomes and complications of OWHTO, (2) morphological and anatomical changes induced by OWHTO, (3) biomechanical studies using multibody or finite element (FE) modeling techniques in relevance to assisting HTO. During the search process, standardized medical subject headings (MeSH terms) including “high tibial osteotomy,” “analysis, finite element,” “medial collateral ligament, knee,” and “articulation, patellofemoral,” and text words including “tibial slope,” “pressure,” “patellar height,” and “patellar tracking” were used. Meaningful combinations of these terms and words were used to form possible search strings, for example, (high tibial osteotomy [MeSH terms]) AND ((pressure [MeSH terms]) OR (medial collateral ligament, knee [MeSH terms])).

Following the initial search steps, the titles of all the search outcomes were assessed, and only peer-reviewed studies were collected. The two review authors (E.E., G.C.) analyzed independently the titles and abstracts of the screened articles. At this step, the articles without any abstract were excluded. A second search for relevant articles was performed within the references cited in the selected articles. References were imported into bibliographic management software, and all duplicates were removed. Then, the review authors read the full texts of the selected articles independently.

### 2.2. Eligibility Criteria

All the articles reporting the biomechanical changes induced by OWHTO were included in the review. Besides, articles on the biomechanical modeling of OWHTO using multibody dynamics and FE methods were included. We excluded all articles on lateral closing high tibial osteotomies, double osteotomies, osteotomies performed to treat knee laxities, computer-assisted surgical methods, plate design, and positioning, technical notes as well as the articles related to the other complications of OWHTO that were not in the interest of the current study. A language filter has also been used to only include articles written in English. The exclusion reasons of the full-text articles that were assessed at the eligibility step are presented in Figure 1.

### 2.3. Data Extraction and Quality Assessment

The qualitative and quantitative data of the articles were extracted independently by two review authors of the study (E.E., G.C.). In case of disagreement, a discussion was made between the two authors. The data extracted from the articles were the title of the study, the authors, the year of publication, and the design of the study. Then, each review author compiled in independent tables the main results concerning tibiofemoral pressures according to the MCL status, changes in tibial slope, changes in patellar height and/or patellar tracking, and biomechanical simulations. To evaluate the methodological quality of the studies included in our data analysis, we used the validated QUACS scale (13 items) for cadaver studies and the STROBE scale (22 items) for clinical studies.

## 3. Results

A total of 38 studies met the inclusion criteria for the systematic review. The PRISMA statement flowchart depicted in Figure 1 shows the number of search results (a total of 3062 articles) and the number of articles that were included or excluded [22]. The 38 included articles were then divided into the defined categories based on their topics and provided results. The defined categories, as well as the number of articles included in each category, are as follows: MCL release (6 articles), posterior tibial slope (14 articles), patellar position (12 articles), and biomechanical simulations (6 articles).

### 3.1. MCL Release

Six articles studying the effect of MCL release on tibiofemoral contact and valgus laxity (Table 1) were included. As presented in Table 1, the alteration in the contact pressure and contact area in the medial and lateral compartments are reported after osteotomy. These results are categorized based on the level of release done on the superficial bundle of MCL (sMCL) and the amount of alignment correction during HTO. Besides, the change in valgus laxity has been reported by three studies. The quality of the studies (QUACS or STROBE scores) has also been assessed based on the nature of the study and reported.

### 3.2. Tibial Slope

Fourteen articles were included in the tibial slope category, and the corresponding results are provided in Table 2. The osteotomy techniques used in these studies vary between conventional (monoplanar) osteotomy (with and without navigation) and biplanar osteotomy. In addition to the posterior tibial slope before and after surgery, the difference of this variable is provided to simplify comparisons between studies. The statistically significant results are marked in red (Table 2).

### 3.3. Patellar Position

Twelve studies were selected for the category of patellar position (Table 3). The reported outputs of the selected studies are divided into patellar height, lateral patellar tilt, and patellar shift. Considering that various methods were used to assess the patellar height in the selected studies, five different indices were chosen to compare the alteration in the patellar height after HTO. These indices include Insall-Salvati, modified Insall-Salvati, Caton-Deschamps, Blackburne-Peel, and Modified Blumensaat as defined in the literature [23, 24]. The results of the quality assessment of the selected papers (STROBE scores) are also presented in Table 3.

### 3.4. Biomechanical Simulations

Among the selected articles in the current review, a total of six articles have chosen a biomechanical simulation approach with generic or subject-specific modeling (Table 4). These articles were mainly focused on testing the effect of the alignment principle on tibiofemoral contact balancing or estimating the optimum alignment based on subject-specific models. One article had studied the effect of MCL slackness and MCL release on the biomechanical outcomes. The objectives, findings, and various validation methods of these studies are presented in Table 4.

## 4. Discussion

### 4.1. MCL Release and Its Correlation with Tibiofemoral Contact Pressure

The MCL is composed of two bundles. The superficial bundle is distally attached to the medial aspect of the proximal part of the tibia and the deep bundle that is attached to the joint capsule. To perform OWHTO, the medial proximal part of the tibia needs to be exposed. As a result, to properly expose this region and based on the condition of MCL in each patient, various strategies might be adopted by the surgeons concerning the MCL: preservation, selective release of the superficial bundle, or a complete release of the superficial bundle. This of course raises concern about the effect of sMCL release on valgus stability and also leads to questioning the correct approach to take concerning sMCL and its effect on the tibiofemoral contact pressures.

As shown in Table 1, various studies showed that performing an OWHTO without any release of the sMCL results in an increase of the sMCL strain, an increase in the contact area and pressures on the medial tibiofemoral compartment, and a decrease in these parameters on the lateral compartment [18, 27, 28]. This condition, which is in contrast with the objective of performing OWHTO, can even be deteriorated by increasing the size of the opened wedge. The results of the cadaveric study performed by Seitz et al. showed that a 5° and 10° wedge opening in the tibia, respectively, increased the medial contact pressure up to 0.11 and 0.14 MPa with respect to the pressure before surgery [18].

Generally, the release of the superficial bundle resulted in a decrease in the contact area and pressures on the medial compartment and an increase in these parameters on the lateral compartment [18, 27, 28]. For instance, for a 10° opening during osteotomy, there was a significant decrease in the medial tibiofemoral pressure after completely releasing sMCL in comparison to the unreleased state [18, 27]. This decrease was reported to be 0.13 MPa by Seitz et al. [18] and 0.17 MPa by Van Egmond et al. [27]. In the same category, Agneskirchner et al. reported an average pressure decrease of 0.44 MPa and 0.64 MPa, respectively, by 50% sMCL release and complete sMCL release, with respect to unreleased sMCL in osteotomies performed to move the mechanical axis of the knee to pass through the Fujisawa point [28]. Although it is important to bear in mind that the actual goal was to reduce the medial contact pressure and contact surface compared to the intact knee, which was not achieved by 50% MCL release as the respective 0.24 MPa and 29.7 mm^2^ increases in these values imply. As concerns the lateral compartment, the results seemed contradictory in many cases. The results provided by Seitz et al. [18] and Agneskirchner et al. [28] showed that the pressure and area of contact after OWHTO has decreased in the lateral compartment regardless of the sMCL release. These results were in contrast with the results of Van Egmond et al. and Suero et al. who reported an increase in these values [27, 29].

As previously mentioned, MCL release could have a negative impact of increasing the valgus laxity that could clinically induce a feeling of instability for the patient. Concerning laxity of the knee during valgus stress, there was less consensus on the outcomes. The study performed by Pape et al. suggested that releasing the sMCL increases the valgus laxity and thus it should be kept to a minimum to decrease the potential of late valgus instability [25]. However, the alignment of the cadaver knees has not been altered in this study, and the conclusion has been made without performing any HTOs. This finding was supported by the study of Van Egmond et al. that showed a laxity increase of nearly 8° after a complete release of the sMCL [27]. On the contrary, the clinical study of Seo et al. [26] revealed that the increase of the medial joint opening (MJO) because of complete release of sMCL was totally recovered after opening the wedge during medial osteotomy. There was no significant difference between the preoperative and postoperative MJO values at 3, 6, and 12 months after surgery.

Most authors seemed to have a consensus that releasing the superficial bundle of the MCL during OWHTO helps with better achieving the goals of the surgery, although complete information about the releasing technique was missing in many cases. Indeed, when no release was performed, the opening of the gap of the osteotomy caused a significant increase in the MCL strain [18] and therefore medial tibiofemoral pressures, whereas, when the release was performed, the medial tibiofemoral pressures dropped significantly. However, from observation of the contradictory results reported in the literature, we can conclude that the different factors that are playing a role in the sMCL tension need to be fully decomposed. Therefore, adding a biomechanical perspective to the sMCL question also seems to be required to acquire a better understanding of this complication such as the study performed by Purevsuren et al. [53]. The sMCL of each patient has a particular preexisting tension in it; this tension is of course reduced by partially releasing the sMCL bundles while performing OWHTO. In addition to this, if we consider that the osteotomy cut is performed superior to the insertion of sMCL, opening the wedge results in retensioning the sMCL relative to the size of the opened wedge [25]. Consequently, the final tension remaining in the sMCL after OWHTO is affected by the amount of release, the size of the opened wedge, and also the preexisting tension in it before surgery. So from a biomechanical perspective, if the patient has a preoperative lax MCL, and if the surgeon partially detaches the sMCL to open a small wedge on the tibia, it is expected that the MCL could end up lax. It is therefore recommended in that case to avoid sMCL release as suggested by Pape et al. [25]. On the other end, if the MCL is not lax preoperatively and if the size of the opened wedge on the tibia is large, the MCL would end up being tight and further sMCL release is required to reduce the medial pressure. In this regard, we can conclude that reporting further details about the preoperative conditions of the patient, such as ligament laxity, could help with interpreting from the cadaveric and clinical studies and thus needs to be considered in the design of future studies on this matter.

### 4.2. Tibial Slope Modification

The traditional planning methods for OWHTO rely on the coronal view imaging data to define the required correction angle [6, 57]. In the planning based on the coronal view, the distal portion of the tibia is rotated around a hinge point. Meanwhile, in 3-dimensions, this hinge point is a hinge axis in the anterior-posterior direction and thus it is seen as a point in the coronal view. However, in practice, the hinge axis is not necessarily in the anterior-posterior direction which means that the tibial slope in the sagittal plane can be modified during OWHTO as described by Noyes et al. [58]. This can cause a change in the kinematics as well as in the stability of the knee. The normal range for the posterior tibial slope is 7° to 10° [59]. An increased posterior tibial slope induced an anterior translation of the tibia with respect to the femur as reported by Giffin et al. [17]. Based on our observation, there was a lack of consensus on whether or not an increased posterior slope can increase the ACL strain and cause a higher risk of rupture and chronic anterior knee laxity. The in situ studies of Shelburne et al. have shown that for a 5° increase in the posterior tibial slope, the ACL strain is increased by 26% [60]. On the other hand, Giffin et al. [17] and Martineau et al. [30] did not observe a significant change in the cruciate ligament forces or strains under the loading conditions of their cadaveric studies.

There were recommendations in the literature that enable the surgeon to maintain the tibial slope that is in the normal range or to correct it during OWHTO. This included the use of the 3-triangle method proposed by Noyes et al. [58] or the tables provided in the study of Hernigou et al. [5]. Besides, other authors have proposed mathematical formulas to achieve a targeted tibial posterior slope [61] or to avoid the changes in a posterior tibial slope while performing an osteotomy [62]. Other than the recommendations for the conventional OWHTO, the use of other surgical methods such as the Biplanar osteotomy has been shown to significantly help with the conservation of the tibial slope as reported by Elmali et al. [35]. Indeed, the use of patient-specific 3D printed guides could also help in this context to conserve or modify the tibial slope so that it lies in the normal range.

Among the 14 selected studies related to the alteration of the posterior tibial slope, eight studies found statistically significant results, and most of them (*n* = 7) show that performing OWHTO can lead to a significant increase in posterior tibial slope. Increases are variable among studies. The meta-analysis performed by Nha et al. found an average of 2° increase after pooling the data of 27 studies with various measurement methods [40]. As this alteration is relatively small, they concluded it may have little effect on the biomechanics of the cruciate ligaments. Higher increase rates were reported by other studies such as the study performed by Ozel et al. [31], who reported a 7° increase in the posterior tibial slope after OWHTO. This 7° increase was a major modification because it increased the tibial slope up to twice its initial value but the authors have found no correlation between the postoperative Lysholm knee scores and the increase in the posterior tibial slope angle. This can imply that the clinical outcome scores might not be completely capable of representing the alterations in the radiographic outcomes such as the posterior slope. This idea was supported by the literature review conducted by Yan et al. [41] to compare the outcomes of navigated HTO and conventional HTO. Despite the significant improvement in the radiographic outcomes using navigation HTO, they have observed that these improvements have not yet been reflected in clinical outcome scores. In this sense, the abilities of simulation-based studies could be useful to further analyze such points in the future and to move towards making patient-specific sMCL release decisions.

### 4.3. Patellar Position Modifications

From the biomechanical perspective, it is expectable that monoplanar OWHTO causes a decrease in patellar height by distalization of the anterior tibial tuberosity which is the insertion of the patellar tendon. Among the studies that were selected in the current review, 11 studies had monitored the patellar height alteration after OWHTO (Table 3). Among the various indices used to assess patellar height, the Blackburne-Peel has been the most popular and has been used by 9 out of 12 studies. The reported Blackburne-Peel ratio has decreased in all these studies with 8 of them reporting statistically significant data, thus, proving the patellar height decrease after conventional OWHTO. However, this type of consensus is lacking about the Insall-Salvati and modified Insall-Salvati indices. Among the seven studies reporting the Insall-Salvati ratio, only three of them have monitored a statistically significant alteration with two of them reporting a decrease and one of them reporting an increase in this ratio for a conventional OWHTO. This lack of consensus as mentioned by Hanada et al. [24] seemed to be related to the fact that the Insall-Salvati ratio shows the length of the patellar tendon and does not necessarily represent the patellar height against the femur. The Blackburne-Peal ratio evaluates the patellar height, but in the context of HTO studies, its eligibility can be questioned because it is dependent on the posterior tibial slope which is itself a variable in HTO. As a result, other indices such as Caton-Deschamps and Modified Blumensaat could be more appropriate. Caton-Deschamps ratio has been used by three studies, and all have reported a significant decrease in patellar height after OWHTO. Modified Blumensaat has been proposed by Hanada et al., and they have shown a significant decrease in the patellar height after OWHTO [24].

Regarding the patellar tilt, four studies have shown significant alterations in the patellar tilt with three of them showing significant decreases in the lateral patellar tilt between 1.8° and 2.2° [23, 46, 48], and one of them reported a significant increase of medial patellar tilt of 2.2° using an MRI-based method [15]. Indeed, the exact clinical effect of alteration in patellar position is still unclear on patellofemoral pain even though symptoms of association with patellofemoral pain have been observed with patellar lateral shift [19]. Meanwhile, with regards to patellar shift, only the D'Entremont et al. found a significant increase of 0.94 mm (*p* < 0.001) compared to the preoperative situation using MRI based method [15]. Given the exact measurement method in that study, the matter of patellar shift shall be further investigated in studies with different methods. A correlation between the patella position and the short and midterm clinical outcomes has not been found [64]; however, patellofemoral arthritis has been observed in second look-arthroscopy after OWHTO [20]. In this sense, the matter of patellar position alteration and its impacts on the patellofemoral joint shall be further investigated in future studies. In addition, the correlation between the wedge size and patellar position alteration was not found in the analyzed literature and can be targeted with a simulation-based biomechanical study.

Performing biplanar osteotomies could reduce patellar position alteration by keeping the tibial tuberosity connected to the proximal fragment. The comparison of OWHTO groups with or without biplanar osteotomy provided further insight. Longino et al. [43] showed a significant difference between the two groups with a decrease of 0.09 of the patellar height in the biplanar osteotomy group against 0.19 in the monoplanar group for the Caton-Deschamps index. Park et al. [23] also found a significantly smaller decrease in modified Blackburne-Peel and Caton-Deschamps for the biplanar versus monoplanar group as the position of the patellar tendon insertion on the tibia is conserved in this surgical method.

### 4.4. Biomechanical Studies

The alignment correction amount is closely correlated to the pressure distribution in the two compartments of the knee. As a result, a series of studies have attempted to find the optimal correction angle through monitoring the stress distribution of the cartilage using FE and multibody modeling techniques. Zheng et al. have proposed a subject-specific modeling procedure to identify the alignment that balances the compressive and shear stresses of the cartilage [65]. A preliminary FE study performed by Martay et al. made a general conclusion and proposed that the safe zone for WBA of the lower limb can be between 50% and 60% of the mediolateral tibial width (0° varus-valgus to 2.6–2.8° valgus) [51]. However, to consider the findings of the aforementioned simulation-based studies to be valid and applicable in the medical field, various points require further investigation. First, the high importance of the soft tissues in maintaining the correction angle in HTO seemed to be almost neglected by ignoring the alteration in ligament tensions after the realignment of the knee and by not considering the preexisting laxities that could be present in the ligaments. This is true both in models that are using simplified axial ligaments [51, 56] or in more advanced studies where the 3D FE representative of the ligaments was present [65]. This was while the results of the multibody study performed by Purevsuren et al. showed that preexisting laxity in MCL has an effect on the contact distribution after HTO [53].

Second, simulating the knee under axial loading conditions in the aforementioned studies was not sufficient for monitoring knee contact pressure and for concluding about the correction angle. This issue was true for other studies such as the one performed by Mootanah et al. [52] who have simulated HTO by applying varus/valgus bending moments. The contact pressure balance between the knee compartments can vary along with the knee flexion range, and since the knee flexes up to 20° during the lean phase of a gait cycle, modeling with a single axial load at the stance phase does not represent the full conditions of the problem. Besides, performing studies that take into account the dynamic aspect of knee function in flexion seems to be required to better investigate the unsatisfactory results of HTO. Third, the validation of the model and, as part of it, the adjustment of the material properties are considered as required steps in patient-specific studies designed to obtain the proper alignment to be used [52]. However, this issue has been undervalued in many of the performed studies with this motivation. As a result, although there is a high potential in using FE studies to assist in redefining the correction angles both in general and patient-specific cases, the existing models with that objective tend to oversimplify the problem. However, these simplified studies with their biomechanical point of view can also play an important role in better distinguishing the involving factors in HTO outcomes and thus better designing the clinical and cadaveric studies.

### 4.5. Limitations

The current systematic literature review suffers from a number of limitations. The searching process was only performed on three data sources, and no article of grey literature was included. Furthermore, a bias could have been present in the selection process due to the selection filters such as the language filter and exclusion of articles without abstract. As it is inherent to the systematic reviews, a publication bias might have appeared with an increased prevalence of articles presenting statistically significant results.

## 5. Conclusion

In the current study, a systematic review of the literature was performed on particular complications of OWHTO with a translational approach that covers a diverse set of articles from clinical and cadaveric studies to model-based biomechanical studies. It was highlighted that a correlation exists between the opened wedge during HTO and surgical complications such as increased posterior tibial slope, patellar height decrease, and MCL tightness. Analyzing these complications from a biomechanical perspective clarified that such complications could be impacted by the exact shape and size of the opened wedge that also alters the insertion of sMCL and patellar tendon. Meanwhile, during the traditional planning and execution steps of OWHTO, the impact of the opened wedge on the sagittal view as well as the alteration of soft tissue insertions is normally neglected. Thus, many of the clinical and cadaveric studies focused on the aforementioned complications tend not to collect and provide information about parameters such as preoperative soft tissue condition, preoperative tibial slope, and preoperative limb alignment. However, further information about these parameters seemed to be necessary to be able to come to a better consensus on the alignment principles and how to avoid these complications. This point shall be considered in the design of future studies on the topic. The ability of biomechanical simulations in isolating the involved parameters can play an important role in this process.

## Figures and Tables

**Figure 1:** PRISMA flow diagram of the search and selection process and the effect of application of inclusion/exclusion criteria.

**Table 1:** Modifications of joint pressures, contact areas according to the state of the medial collateral ligament. sMCL: superficial MCL; MJO: medial joint opening; ^∗^: statistically significant data.

Authors (year)	Study	No. knees	sMCL release state	Correction amount	Medial contact pressure change from intact state (MPa)	Medial contact area change from intact state (mm^2^)	Lateral contact pressure change from intact state (MPa)	Lateral contact area change from intact state (mm^2^)	Valgus laxity	Comments/highlights	QUACS scale	STROBE
Pape et al. (2006) [25]	Cadaveric	20	Complete release	0°	—	—	—	—	↑ 38% MJO	No HTO performed, the release of sMCL should be kept to a minimum to decrease the potential of late valgus instability especially in patients with small wedge sizes and preexisting	11/13	—
			Anterior bundles release						↑ 39% MJO			

Seo et al. (2016) [26]	Clinical	54	Complete release	Fujisawa point	—	—	—	—	↑ 0.2 mm MJO intra-operative	Medial laxity induced by complete sMCL release can be recovered by opening the osteotomy site.	—	18/22

Van Egmond et al. (2017) [27]	Cadaveric	7	No release	10°	↑0.17∗	↑132.9∗	↓0.02∗	↓47.0	↓0.1°	Release of sMCL helps reducing medial cartilage pressure but significantly increases valgus laxity. Considerable relaxation of MCL over time	9/13	—
			Complete release		0.0∗	↑9.6∗	↑0.01∗	↑7.7	↑7.9°			

Seitz et al. (2018) [18]	Cadaveric	6	No release	5°	↑ 0.11	↑ 9	↓ 0.14	↓ 35	—	For the extended knee, biplanar osteotomy, medial contact pressure decreased most when with 10° correction and releasing MCL	9/13	—
				10°	↑ 0.14	↑ 43	↓ 0.25	↓ 85				
			Complete release	0°	↓ 0.03	↓ 79	↓ 0.24	↓ 97				
				5°	↓ 0.05	↓ 63	↓ 0.11	↓ 35				
				10°	↑ 0.01	↓ 125	↓ 0.14	↓ 52				

Agneskirchner et al. (2007) [28]	Cadaveric	6	No release	9 mm	↑ 0.68 ∗	↑ 78.4	↓ 0.3 ∗	↓ 91.7	—	Under 1000 N load passing from 62% valgus position (the effect of different loading axes has also been studied for the intact knee), biplanar osteotomy, high medial pressure maintains despite shifting the loading axis into valgus, decompression happens only after complete release of MCL distal fibers.	9/13	—
			50% release		↑ 0.24 ∗	↑ 29.7	↓ 0.24 ∗	↓ 35.2				
			Complete release		↓ 0.04 ∗	↓ 15.0	↓ 0.08 ∗	↓ 47.7				

Suero et al. (2015) [29]	Cadaveric	7	Complete release	5°	↑ 3% ∗	↑ 9%	↑ 33%	↑ 11%	—	Under 550 N axial load, we have only reported the percentage of alterations in the contact pressure and contact area. The reason for this decision was that the reported values were not consistent with the other studies although the units were the same.	11/13	—
				10°	↓ 23%	↓ 21%	↑ 84%	0%				
				15°	↓ 64%	↓ 46%	↑ 141%	↓ 2%				

**Table 2:** Modifications of the tibial slope. PTS: posterior tibial slope; HTO: high tibial osteotomy; HKA: standing hip–knee–ankle; OW: open-wedge; CW: closed-wedge; ^∗^: statistically significant data.

Authors (year)	Study type	Osteotomy technique		No. knees	Correction amount	PTS pre-HTO	PTS post-HTO	PTS difference	QUACS	STROBE
Martineau et al. (2010) [30]	Cadaveric	OW		6	5 mm	8°	12.1°	↑ 4.1° ∗	7/13	
					10 mm		16.3°	↑ 8.3° ∗		

Ozel et al. (2017) [31]	Clinical	OW		39	Mean HKA 183.7°	8°	15°	↑ 7° ∗		14/22

Sterett et al. (2009) [32]	Clinical	OW		82	—	12.5°	16.5°	↑4° ∗		18/22

Lee et al. (2014) [33]	Clinical	OW	With navigation	40	Fujisawa point	10.5°	11.5°	↑1°		17/22
			Without navigation	40		8.7°	8.2°	↓0.5°		

Nerhus et al. (2017) [34]	Clinical	OW (CW studied but not reported here)		70 total	HKA 186°	7°	8°	↑1° ∗		17/22

Noyes et al. (2006) [4]	Clinical	OW		55	—	9°	10°	↑1°		15/22

Elmali et al. (2013) [35]	Clinical	OW	Monoplanar osteotomy	56	HKA 186.4	10.1°	11.7°	↑1.6° ∗		15/22
			Biplanar osteotomy	32	HKA 185.4	9.9°	10.7°	↑0.8° ∗		

Birmingham al. (2009) [36]	Clinical	OW		126	HKA 180°	5.15°	6.37°	↑1.22° ∗		15/22

Chang et al. (2017) [37]	Clinical	OW	With navigation	41	WBA passing 64.3%	11.7°	12.2°	↑0.5°		19/22
			Without navigation	66	WBA passing 57.3%	12.1°	13.1°	↑1°		

Na et al. (2018) [38]	Clinical	OW		71	HKA: 182.6° (varus > 4°)	10.6° (varus > 4°)	10.9° (varus > 4°)	↑0.3° (varus > 4°)		18/22
					HKA: 184.2° (varus < 4°)	10.0° (varus < 4°)	10.7° (varus < 4°)	↑0.7° (varus < 4°)		

Van Egmond et al. (2016) [39]	Cadaveric	OW (CW studied but not reported here)		25 OW	HKA: 184.3° (open)	—	16.2° (open)	↑1.6°	9/13	

Nha et al. (2016) [40]	Clinical meta-analysis	OW (CW studied but not reported here)		—	—	—	—	↑2° ∗		

Yan et al. (2016) [41]	Literature review	OW	With navigation	1608	—	Navigated HTO produces significantly less change in PTS compared to conventional methods.				
			Without navigation	608						

Wu et al. (2017) [42]	Comprehensive meta-analysis	OW and CW		663 OW 581 CW	—	Open-wedge HTO showed greater PTS angle compared to closed-wedge, ↑1.31° ∗				

**Table 3:** Patellar position modifications during OWHTO. NS: not significant; ^∗^: statistically significant data; mBP: modified Blackburne-Peel ratio; OW: open-wedge; Clin.: clinical study; Monopl.: monoplanar; Postop.: postoperative.

Authors (year)	Study type	Osteotomy technique		No. knees	Correction amount	Patellar height					Lateral tilt	Shift (mm)	STROBE
						Insall-Salvati	Modified Insall-Salvati	Caton-Deschamps	Blackburne-Peel	Modified Blumensaat			
Longino et al. (2013) [43]	Clin.	OW	Biplanar	29	HKA: 180.8°	—	—	↓0.09∗	↓0.10∗	—	—	—	19/22
			Monopl.	29	HKA: 179.9°	NS	NS	↓0.19∗	↓0.23∗	—	—	—	

Hanada et al. (2014) [24]	Clin.	OW (CW not reported here)		10	WBA passing 62.5%	↑0.308∗ (postop.) ↑0.238 (NS) (after 1 year)	—	—	—	↓ 0.094∗ (postop.) ↓0.153∗ (after 1 year)	—	—	13/22

Tanaka et al. (2018) [44]	Clin.	Biplanar OW		52	HKA: 181.3°	—	—	↓0.16∗	—	—	—	—	14/22

Park et al. (2017) [23]	Clin.	OW	Biplanar	33	HKA: 180.3°	↓0.01	↑0.01	↓0.04∗	↓0.03∗	—	↓1.40°∗	↓0.01	16/22
			Monopl.	30	HKA: 180.8°	↓0.05∗	↓0.08∗	↓0.10∗	↓0.09∗		↓2.00°∗	↓0.01	

Fan (2012) [45]	Clin.	OW		9	HKA: 183.9°	↑0.07	—	—	↓0.19∗	—	—	—	10/22

Bito et al. (2010) [46]	Clin.	OW		49	—	—	—	—	mBP ↓0.2∗	—	↓2.2°∗	NS	11/22

Song et al. (2012) [47]	Clin.	OW (CW not reported here)		50	—	—	—	—	↓0.10∗	—	↑0.6°	↑0.4	9/22

Lee et al. (2016) [48]	Clin.	OW		46	HKA: 181.4°	—	—	—	↓0.1∗	—	↓1.8°∗	NS	11/22

D'Entremont et al. (2014) [15]	Clin.	OW		14	—	—	—		—	—	↓2.20°∗	↑0.9∗	17/22

Birmingham et al. (2009) [36]	Clin.	OW		126	HKA: 180°	NS	—	—	↓0.05∗	—	—	—	15/22

Elmali et al. (2013) [35]	Clin.	OW	Biplanar	32	HKA: 185.4°	NS	—	—	NS	—	—	—	15/22
			Monopl.	56	HKA: 186.4°	↓0.07∗	—	—	↓0.07∗	—	—	—	

Noyes et al. (2006) [4]	Clin.	OW		55	—	—	—	—	↓0.09	—	—	—	15/22

**Table 4:** Biomechanical studies on the OWHTO alignment and related surgical complications. PTS: posterior tibial slope; OW: open-wedge; CW: closed-wedge.

Authors (year)	Simulation technique	Osteotomy technique	Ligament modeling	Loading condition	Objective	Outcomes	Validation method
Zheng et al. [65]	FE	OW	3D FE	Subject-specific loading data at 5% of the gait cycle obtained from gait analysis	Introducing a subject-specific modeling procedure to see the biomechanical effects of HTO alignment on tibiofemoral cartilage stress distribution.	Providing a platform for noninvasive, patient-specific preoperative planning of the osteotomy	Maximum contact pressure was compared to literature under similar axial loading [49, 50]

Martay et al. (2017) [51]	FE	OW	Axial	Loading and alignment calculated from motion analysis data at the point of maximum load in the walking cycle	How different WBA realignments affected load distribution in the knee, to find the optimal postsurgical realignment.	Proposing a new target for WBA correction being 55% tibial width (1.7°–1.9° valgus),	Validated their model creation method using porcine specimens. Compared their HTO related results to a published human cadaveric study [52].

Purevsuren et al. (2019) [53]	Multi-body dynamics	OW	Axial	Axial load in standing position	Effects of MCL laxity, loading axis correction, and different types of MCL release, on the medial-lateral contact force distribution after OWHTO Determining the necessary MCL release strategy for balanced load distribution	MCL slackness affected load distribution of the knee after HTO. Anterior and middle bundle release shown to be the optimal surgical method to balance contact distribution in simulated standing position. Only anterior bundle release is recommended for knees with a large amount of MCL slackness. No effect observed by changing the simulated axis correction.	Compared estimated medial and lateral contact distribution after HTO with previous cadaveric studies [28, 54].

Mootanah et al. (2014) [52]	FE	None	3D FE (tuned to minimize kinematic difference from cadaver specimen)	Axial load + varus and valgus bending moments (0 to 15 nm) applied about the knee joint center to simulate different malalignment degrees	Predicting knee joint contact forces and pressures for different degrees of malalignment.	Generated knee model could give an accurate prediction of normalized intra-articular pressure and forces for different loading conditions. The model could be further developed for subject-specific surgical planning.	Cadaveric study performed having matching boundary and loading conditions.

Kuriyama et al. (2019) [55]	Dynamic musculo-skeletal modeling	OW	Axial	Gait and squat	Determining the ideal coronal alignment under dynamic conditions	Approved the validity of classical target alignment. Over-correction should be avoided. Increased PTS caused excessive ACL tightness due to femoral posterior positioning with respect to tibia. PTS increase resulted in LCL tightness and PCL and MCL laxity.	Comparing the kinematics of the native knee model with the in vivo kinematics obtained from a healthy volunteer.

Trad et al. (2018) [56]	FE	CW	Axial	Axial load in standing position	Effect of varying the high tibial osteotomy correction angle on the stress distribution in two tibiofemoral compartments Finding the optimal correction angle to achieve a balanced loading between compartments.	Achieving a balanced stress distribution in two compartments and desired alignment under a valgus hypercorrection of 4.5 degrees Study findings agree well with clinical data and recommendations found in the literature [8].	Compared against experimental and numerical results from the literature. CW article included as it concerns alignment principle.

## Data Availability

The data used to support the findings of this study are included within the article.

## References

[1] Agarwala S., Sobti A., Naik S., Chaudhari S. (2016). Comparison of closing-wedge and opening-wedge high tibial osteotomies for medial compartment osteoarthritis of knee in Asian population: mid-term follow-up. *Journal of Clinical Orthopaedics and Trauma*.

[2] Duivenvoorden T., Brouwer R. W., Baan A. (2014). Comparison of closing-wedge and opening-wedge high tibial osteotomy for medial compartment osteoarthritis of the Knee. *Journal of Bone and Joint Surgery*.

[3] Loia M. C., Vanni S., Rosso F. (2016). High tibial osteotomy in varus knees: indications and limits. *Joints*.

[4] Noyes F. R., Mayfield W., Barber-Westin S. D., Albright J. C., Heckmann T. P. (2006). Opening wedge high tibial Osteotomy. *The American Journal of Sports Medicine*.

[5] Hernigou P., Medevielle D., Debeyre J., Goutallier D. (1987). Proximal tibial osteotomy for osteoarthritis with varus deformity. A ten to thirteen-year follow-up study. *The Journal of Bone & Joint Surgery*.

[6] Dugdale T. W., Noyes F. R., Styer D. (2007). Preoperative planning for high tibial osteotomy. *Clinical Orthopaedics and Related Research*.

[7] Koshino T., Tsuchiya K., Shiomi S. (1979). The effect of high tibial osteotomy on osteoarthritis of the knee. *The Orthopedic Clinics of North America*.

[8] Hernigou P., Ovadia H., Goutallier D. (1992). Mathematical modelling of open-wedge tibial osteotomy and correction tables. *Revue de Chirurgie Orthopédique et Réparatrice de l'Appareil Moteur*.

[9] Insall J. N., Joseph D. M., Msika C. (1984). High tibial osteotomy for varus gonarthrosis. A long-term follow-up study. *The Journal of Bone and Joint Surgery. American Volume*.

[10] DeMeo P. J., Johnson E. M., Chiang P. P., Flamm A. M., Miller M. C. (2010). Midterm follow-up of opening-wedge high tibial osteotomy. *The American Journal of Sports Medicine*.

[11] Sprenger T. R., Doerzbacher J. F. (2003). Tibial osteotomy for the treatment of varus GONARTHROSIS. *The Journal of Bone and Joint Surgery. American Volume*.

[12] Benzakour T., Hefti A., Lemseffer M., Ahmadi J. D., Bouyarmane H., Benzakour A. (2010). High tibial osteotomy for medial osteoarthritis of the knee: 15 years follow-up. *International Orthopaedics*.

[13] Mina C., Garrett W. E., Pietrobon R., Glisson R., Higgins L. (2008). High tibial osteotomy for unloading osteochondral defects in the medial compartment of the knee. *The American Journal of Sports Medicine*.

[14] Briem K., Ramsey D. K., Newcomb W., Rudolph K. S., Snyder-Mackler L. (2007). Effects of the amount of valgus correction for medial compartment knee osteoarthritis on clinical outcome, knee kinetics and muscle co-contraction after opening wedge high tibial osteotomy. *Journal of Orthopaedic Research*.

[15] d’Entremont A. G., McCormack R. G., Horlick S. G. D., Stone T. B., Manzary M. M., Wilson D. R. (2014). Effect of opening-wedge high tibial osteotomy on the three-dimensional kinematics of the knee. *The Bone & Joint Journal*.

[16] Martin R., Birmingham T. B., Willits K., Litchfield R., Lebel M. E., Giffin J. R. (2014). Adverse event rates and classifications in medial opening wedge high tibial osteotomy. *The American Journal of Sports Medicine*.

[17] Giffin J. R., Vogrin T. M., Zantop T., Woo S. L.-Y., Harner C. D. (2004). Effects of increasing tibial slope on the biomechanics of the knee. *The American Journal of Sports Medicine*.

[18] Seitz A. M., Nelitz M., Ignatius A., Dürselen L. (2019). Release of the medial collateral ligament is mandatory in medial open-wedge high tibial osteotomy. *Knee Surgery, Sports Traumatology, Arthroscopy*.

[19] MacIntyre N. J., Hill N. A., Fellows R. A., Ellis R. E., Wilson D. R. (2006). Patellofemoral joint kinematics in individuals with and without patellofemoral pain syndrome. *The Journal of Bone & Joint Surgery*.

[20] Kim K.-I., Kim D. K., Song S. J., Lee S. H., Bae D. K. (2017). Medial open-wedge high tibial osteotomy may adversely affect the patellofemoral joint. *Arthroscopy: The Journal of Arthroscopic & Related Surgery*.

[21] McGowan J., Sampson M., Salzwedel D. M., Cogo E., Foerster V., Lefebvre C. (2016). PRESS peer review of electronic search strategies: 2015 guideline statement. *Journal of Clinical Epidemiology*.

[22] Moher D., Liberati A., Tetzlaff J., Altman D. G., The PRISMA Group (2009). Preferred reporting items for systematic reviews and meta-analyses: the PRISMA statement. *PLoS Medicine*.

[23] Park H., Kim H. W., Kam J. H., Lee D. H. (2017). Open wedge high tibial osteotomy with distal tubercle osteotomy lessens change in patellar position. *BioMed Research International*.

[24] Hanada M., Takahashi M., Koyama H., Matsuyama Y. (2014). Comparison of the change in patellar height between opening and closed wedge high tibial osteotomy: measurement with a new method. *European Journal of Orthopaedic Surgery and Traumatology*.

[25] Pape D., Duchow J., Rupp S., Seil R., Kohn D. (2006). Partial release of the superficial medial collateral ligament for open-wedge high tibial osteotomy. *Knee Surgery, Sports Traumatology, Arthroscopy*.

[26] Seo S.-S., Kim C.-W., Seo J.-H., Kim D.-H., Lee C.-R. (2016). Does superficial medial collateral ligament release in open-wedge high tibial osteotomy for varus osteoarthritic knees increase valgus laxity?. *The American Journal of Sports Medicine*.

[27] van Egmond N., Hannink G., Janssen D., Vrancken A. C., Verdonschot N., van Kampen A. (2017). Relaxation of the MCL after an open-wedge high tibial osteotomy results in decreasing contact pressures of the knee over time. *Knee Surgery, Sports Traumatology, Arthroscopy*.

[28] Agneskirchner J. D., Hurschler C., Wrann C. D., Lobenhoffer P. (2007). The effects of valgus medial opening wedge high tibial osteotomy on articular cartilage pressure of the knee: a biomechanical study. *Arthroscopy: The Journal of Arthroscopic & Related Surgery*.

[29] Suero E. M., Sabbagh Y., Westphal R. (2015). Effect of medial opening wedge high tibial osteotomy on intraarticular knee and ankle contact pressures. *Journal of Orthopaedic Research*.

[30] Martineau P. A., Fening S. D., Miniaci A. (2010). Anterior opening wedge high tibial osteotomy: the effect of increasing posterior tibial slope on ligament strain. *Canadian Journal of Surgery*.

[31] Ozel O., Yucel B., Mutlu S., Orman O., Mutlu H. (2017). Changes in posterior tibial slope angle in patients undergoing open-wedge high tibial osteotomy for varus gonarthrosis. *Knee Surgery, Sports Traumatology, Arthroscopy*.

[32] Sterett W., Miller B., Joseph T., Rich V., Bain E. (2009). Posterior tibial slope after medial opening wedge high tibial osteotomy of the varus degenerative knee. *The Journal of Knee Surgery*.

[33] Lee D.-H., Han S.-B., Oh K.-J. (2014). The weight-bearing scanogram technique provides better coronal limb alignment than the navigation technique in open high tibial osteotomy. *The Knee*.

[34] Nerhus T. K., Ekeland A., Solberg G., Sivertsen E. A., Madsen J. E., Heir S. (2017). Radiological outcomes in a randomized trial comparing opening wedge and closing wedge techniques of high tibial osteotomy. *Knee Surgery, Sports Traumatology, Arthroscopy*.

[35] Elmali N., Esenkaya I., Can M., Karakaplan M. (2013). Monoplanar versus biplanar medial open-wedge proximal tibial osteotomy for varus gonarthrosis: a comparison of clinical and radiological outcomes. *Knee Surgery, Sports Traumatology, Arthroscopy*.

[36] Birmingham T. B., Giffin J. R., Chesworth B. M. (2009). Medial opening wedge high tibial osteotomy: a prospective cohort study of gait, radiographic, and patient-reported outcomes. *Arthritis Care and Research*.

[37] Chang J., Scallon G., Beckert M. (2017). Comparing the accuracy of high tibial osteotomies between computer navigation and conventional methods. *Computer Assisted Surgery*.

[38] Na Y., Lee B., Hwang D., Choi E., Sim J. A. (2018). Can osteoarthritic patients with mild varus deformity be indicated for high tibial osteotomy?. *The Knee*.

[39] van Egmond N., van Grinsven S., van Loon C. J. M., Gaasbeek R. D., van Kampen A. (2016). Better clinical results after closed- compared to open-wedge high tibial osteotomy in patients with medial knee osteoarthritis and varus leg alignment. *Knee Surgery, Sports Traumatology, Arthroscopy*.

[40] Nha K.-W., Kim H.-J., Ahn H.-S., Lee D.-H. (2016). Change in posterior tibial slope after open-wedge and closed-wedge high tibial osteotomy. *The American Journal of Sports Medicine*.

[41] Yan J., Musahl V., Kay J., Khan M., Simunovic N., Ayeni O. R. (2016). Outcome reporting following navigated high tibial osteotomy of the knee: a systematic review. *Knee Surgery, Sports Traumatology, Arthroscopy*.

[42] Wu L., Lin J., Jin Z., Cai X., Gao W. (2017). Comparison of clinical and radiological outcomes between opening-wedge and closing-wedge high tibial osteotomy: a comprehensive meta-analysis. *PLoS One*.

[43] Longino P. D., Birmingham T. B., Schultz W. J., Moyer R. F., Giffin J. R. (2013). Combined tibial tubercle osteotomy with medial opening wedge high tibial osteotomy minimizes changes in patellar Height. *The American Journal of Sports Medicine*.

[44] Tanaka T., Matsushita T., Miyaji N. (2019). Deterioration of patellofemoral cartilage status after medial open-wedge high tibial osteotomy. *Knee Surgery, Sports Traumatology, Arthroscopy*.

[45] Fan J. C. H. (2012). Open wedge high tibial osteotomy: cause of patellar descent. *Journal of Orthopaedic Surgery and Research*.

[46] Bito H., Takeuchi R., Kumagai K. (2010). Opening wedge high tibial osteotomy affects both the lateral patellar tilt and patellar height. *Knee Surgery, Sports Traumatology, Arthroscopy*.

[47] Song I. H., Song E. K., Seo H. Y., Lee K. B., Yim J. H., Seon J. K. (2012). Patellofemoral Alignment and Anterior Knee Pain After Closing- and Opening- Wedge Valgus High Tibial Osteotomy. *Arthroscopy: The Journal of Arthroscopic & Related Surgery*.

[48] Lee Y. S., Lee S. B., Oh W. S., Kwon Y. E., Lee B. K. (2016). Changes in patellofemoral alignment do not cause clinical impact after open-wedge high tibial osteotomy. *Knee Surgery, Sports Traumatology, Arthroscopy*.

[49] Peña E., Calvo B., Martínez M. A., Palanca D., Doblaré M. (2005). Finite element analysis of the effect of meniscal tears and meniscectomies on human knee biomechanics. *Clinical biomechanics*.

[50] Haut Donahue T. L., Hull M. L., Rashid M. M., Jacobs C. R. (2002). A finite element model of the human knee joint for the study of tibio-femoral contact. *Journal of Biomechanical Engineering*.

[51] Martay J. L., Palmer A. J., Bangerter N. K. (2018). A preliminary modeling investigation into the safe correction zone for high tibial osteotomy. *The Knee*.

[52] Mootanah R., Imhauser C. W., Reisse F. (2014). Development and validation of a computational model of the knee joint for the evaluation of surgical treatments for osteoarthritis. *Computer Methods in Biomechanics and Biomedical Engineering*.

[53] Purevsuren T., Khuyagbaatar B., Kim K., Kim Y. H. (2019). Effects of medial collateral ligament release, limb correction, and soft tissue laxity on knee joint contact force distribution after medial opening wedge high tibial osteotomy: a computational study. *Computer Methods in Biomechanics and Biomedical Engineering*.

[54] Ogden S., Mukherjee D. P., Keating M. E., Ogden A. L., Albright J. A., McCall R. E. (2009). Changes in load distribution in the knee after opening-wedge or closing-wedge high tibial osteotomy. *The Journal of Arthroplasty*.

[55] Kuriyama S., Watanabe M., Nakamura S. (2020). Classical target coronal alignment in high tibial osteotomy demonstrates validity in terms of knee kinematics and kinetics in a computer model. *Knee Surgery, Sports Traumatology, Arthroscopy*.

[56] Trad Z., Barkaoui A., Chafra M., Tavares J. M. R. (2018). Finite element analysis of the effect of high tibial osteotomy correction angle on articular cartilage loading. *Proceedings of the Institution of Mechanical Engineers, Part H: Journal of Engineering in Medicine*.

[57] Miniaci A., Ballmer F. T., Ballmer P. M., Jakob R. P. (1989). Proximal tibial Osteotomy. *Clinical Orthopaedics and Related Research*.

[58] Noyes F. R., Goebel S. X., West J. (2005). Opening wedge tibial osteotomy: the 3-triangle method to correct axial alignment and tibial slope. *The American Journal of Sports Medicine*.

[59] Brazier J., Migaud H., Gougeon F., Cotten A., Fontaine C., Duquennoy A. (1996). Evaluation of methods for radiographic measurement of the tibial slope. A study of 83 healthy knees. *Revue de Chirurgie Orthopédique et Réparatrice de l'Appareil Moteur*.

[60] Shelburne K. B., Kim H.-J., Sterett W. I., Pandy M. G. (2011). Effect of posterior tibial slope on knee biomechanics during functional activity. *Journal of Orthopaedic Research*.

[61] Lee Y. S., Park S. J., Shin V. I., Lee J. H., Kim Y. H., Song E. K. (2010). Achievement of targeted posterior slope in the medial opening wedge high tibial osteotomy: a mathematical approach. *Annals of Biomedical Engineering*.

[62] Sariali E., Catonne Y. (2009). Modification of tibial slope after medial opening wedge high tibial osteotomy: clinical study and mathematical modelling. *Knee Surgery, Sports Traumatology, Arthroscopy*.

[63] Nha K.-W., Kim H.-J., Ahn H.-S., Lee D.-H. (2016). Change in posterior tibial slope after open-wedge and closed-wedge high tibial osteotomy. *The American Journal of Sports Medicine*.

[64] Goshima K., Sawaguchi T., Shigemoto K., Iwai S., Nakanishi A., Ueoka K. (2017). Patellofemoral Osteoarthritis Progression and Alignment Changes after Open- Wedge High Tibial Osteotomy Do Not Affect Clinical Outcomes at Mid-term Follow-up. *Arthroscopy: The Journal of Arthroscopic & Related Surgery*.

[65] Zheng K., Scholes C. J., Chen J., Parker D., Li Q. (2017). Multiobjective optimization of cartilage stress for non-invasive, patient- specific recommendations of high tibial osteotomy correction angle - a novel method to investigate alignment correction. *Medical Engineering & Physics*.

